# The Novel Tumor Suppressor Gene ZNF24 Induces THCA Cells Senescence by Regulating Wnt Signaling Pathway, Resulting in Inhibition of THCA Tumorigenesis and Invasion

**DOI:** 10.3389/fonc.2021.646511

**Published:** 2021-05-31

**Authors:** Juan Xiong, Panpan Jiang, Li Zhong, Youling Wang

**Affiliations:** ^1^ School of Public Health, Health Science Center, Shenzhen University, Shenzhen, China; ^2^ School of Life and Marine Sciences, Shenzhen University, Shenzhen, China; ^3^ Shenzhen RealOmics (Biotech) Co., Ltd., Shenzhen, China

**Keywords:** ZNF24, thyroid cancer, Wnt signaling pathway, senescence, tumor suppressor genes

## Abstract

**Object:**

Clinically, the effective treatment options available to thyroid cancer (THCA) patients are very limited. Elucidating the features of tumor suppressor genes (TSGs) and the corresponding signal transduction cascade may provide clues for the development of new strategies for targeted therapy of THCA. Therefore, this paper aims to explore the mechanism of ZNF24 underlying promoting THCA cell senescence at molecular level.

**Methods:**

We performed RT-PCR and Western Blotting for evaluating associated RNA and protein expression. CCK8, colony forming, wound healing and Transwell chamber assays were conducted to examine THCA cell proliferation, invasion and migration. β-galactosidase staining assay was performed to detect THCA cells senescence. The size and volume of xenotransplanted tumors in nude mice are calculated to asses ZNF24 effect *in vivo*.

**Results:**

Ectopic expression of ZNF24 significantly inhibited the cell viability, colony forming, migration and invasion abilities of THCA cell lines (K1/GLAG-66i and BCPAPi) (*P* < 0.05). ZNF24 induced BCPAPi cells senescence through regulating Wnt signaling pathway. ZNF24 inhibited Wnt signaling pathway activition by competitively binding β-catenin from LEF1/TCF1-β-catenin complex. In nude mice, both Ectopic expression of ZNF24 and 2,4-Da (the strong β-catenin/Tcf-4 inhibitor) treatment significantly decreased both the size and weight of xenotransplanted tumors when compared with control mice (*P* < 0.05).

**Conclusion:**

Results obtained *in vivo* and *in vitro* reveal the role of ZNF24 in significantly suppressing THCA tumorigenesis and invasion by regulating Wnt signaling pathway.

## Introduction

Thyroid cancer (THCA) accounts for around 90% and 2.5% of endocrine cancers and all cancers, respectively (1). THCA has a three-fold increase incidence among females aged 25 to 65 years than ordinary people (2). The incidence of THCA shows a 4.5% increase annually within the last 10 years, possibly due to improvements in diagnostic technology, Environment (such as radiation, pollution) and lifestyle changes (3). Although progress has been made in various treatments, including immunotherapy, the prognosis of THCA patients is still frustrating. The difficulty in the treatment of THCA patients lies in the restricted knowledge on the tumor occurrence mechanism at molecular level, and it becomes a new research direction over the past few years. Certain intracellular signal transduction pathways are known to be closely related to THCA, including RTK, MAPK, PI3K, and Wnt/β-catenin pathways (4–7).

Wnt signaling pathway related factors including CTNNB1, AXIN1 and APC genes mutations are the markers of poorly differentiated THCA, especially ATC (8). CTNNB1 mutations have been frequently seen (>60%) (9, 10). With the dedifferentiation of THCA, these changes become more frequent (25% in PDTC, 60–65% in ATC) (5). This indicates that CTNNB1 may be closely related to the tumorigenesis of THCA. In addition, Lu et al. have reported that GATA4 directly binds and inhibits the β-catenin activity in transcribing target genes involved in the classical Wnt pathway, which result in Hepatocellular carcinoma (HCC) cells senescence (11). We therefore hypothesize that β-catenin might also be related to THCA tumor cell senescence.

ZNF24, zinc finger transcription factor 24, has been poorly studies so far. Liu et al. suggested the effect of ZNF24 on inhibiting gastric cancer tumor cell invasion and migration (12). In addition, zinc finger transcription factor 191 affects the proliferation of HCC by regulating the Wnt signaling pathway in HCC (13). This implies that ZNF24 may also be related to THCA, and there is a high probability that it will exist as a new type of TSG (tumor suppressor gene). Through analysis of THCA data in TCGA, we found that ZNF24 expression is remarkably high in THCA para-tumoral tissues but low in THCA tumor tissues. Ectopically expressed ZNF24 significantly inhibited cell viability, colony forming, migration and invasion abilities of THCA cells. According to our results, ZNF24 was identified as a tumor suppressor gene not detected in THCA before, which provided a chance to treat ZNF24-deficient THCA cases.

## Materials and Methods

### Ethics Statement

Twenty 4-week-old BALB/Cnu/nu nude mice (20 g) were purchased from Beijing Vital River Laboratory Animal Technology Co., Ltd. and housed in a pathogen-free environment. All experimental protocols were approved by the Institutional Committee for Animal Care and Use at Shenzhen University. All animal work was performed in accordance with the approved protocol.

The protocol for collecting patient samples was approved by Shenzhen University. Written consent was obtained from every patient attending this study. All work was performed in accordance with the approved protocol.

### Reagent

PBS, fetal bovine serum (FBS), DMEM, RPMI medium1640, DMEM/F12 medium and penicillin were brought from GE™ Hyclone company. Cell Signaling Senescence β-Galactosidase Staining Kit was provided by CST company. Doxycycline hyclate were brought from Sigma company; Cell Counting Kit-8 (CCK8) were brought from Dojindo Molecular Technologies company; Lipofectamine™ RNAiMAX transfection reagent was brought from Invitrogen; Antibodies: anti-β-actin (ab8227), anti-β-catenin (ab32503), anti-cMYC (ab71676), anti-CCND2 (ab78612), anti-C-Jun (ab15475), anti-Bcl-2 (ab32124), anti-TCF1 (ab188865), anti-GAPDH (ab76523), Anti-ZNF24(ab254636), anti-LEF1(ab2324), anti-LEF1(ab2324), anti-COX2 (ab15191), anti-MMP2 (ab97779), and anti-MMP9 (ab38898) were purchased from Abcam Co., Ltd, Cambridge, UK. In addition, the working concentration of these primary antibodies is 1 to 2 µg/ml.

### Cell Culture

K1/GLAG-66 cells and BCPAP cells were were obtained from the Cell Bank of Type Culture Collection of Chinese Academy of Sciences (Shanghai, China) and maintained in DMEM/F12 medium (K1/GLAG-66) or RPMI medium1640 (BCPAP) containing 10% FBS (SH30087.01, Hyclone), penicillin (100 U/ml, SH30010, Hyclone) and streptomycin (100 mg/ml), under humid. 37°C, and 5% CO_2_ conditions.

### Generation of Engineered Cell Lines

24 h before transfection, HEK293 cells were transfer into Opti-MEM culture medium. The pMD2.G and psPAX2 packaging plasmids and the pLVX-TetOne-Puro vector constructs for expressing ZNF24 or β-catenin overexpression vector were transfected into HEK293 cells to silence expression using Lipofectamine 2000 (Cat.No.11668019, Invitrogen) in accordance with specific protocols. In brief, vector was diluted with 100 μl Opti-MEM, as called fluid A. Fluid B was Opti-MEM contained 1 µl of Lipofectamine 2000, and dissolved for 5 min before mixed with fluid A. Transfection reagent was added into HEK293 cells were plated in 24-well plates (Cat.No.3548, CORNING). After 4 to 6 h of reaction, culture medium was changed into DMEM full culture medium. After filtering, we utilized the medium that contained recombinant virus for cell infection with 8 µg/ml polybrene. Then, we chosen those affected cells using 0.5 µg/ml puromycin for 7 days prior to later experiments.

### Real-Time PCR

Trizol reagent (#15596018) (Life Technologies, USA) was used to extract total cellular mRNA and then reversed transcribed by the QuantiTect Reverse Transcription Kit (#205313) (Qiagen, Shanghai, China). StepOnePlus system (Applied Biosystem, USA) was utilized to carry out real-time PCR by the use of Thermo Fisher Scientific Maxima SYBR Green/ROX qPCR Master Mix assay (2×) (#K0221). In addition, the BioRad CFX Connect Real-time PCR machine (Bio-rad) and Universal SYBR green reagent were adopted for real-time PCR based on the previous study (14). GAPDH and U6 were used as endogenous reference. Primer sequences used in this study were shown below.

ZNF24-Forward: GTGACAGTGCTGGAGGATTTGG
ZNF24- Reverse: GGTTCTCCACAGCATCAAGCTC
AXIN2-Forward: AAATAACCCCTCAGAGCGATG
AXIN2-Reverse: TTCCAGTTCCTCTCAGCAATC
CCND2-Forward: ACTTGTGATGCCCTGACTG
CCND2-Reverse: ACTTGGATCCGTCACGTTG
c-JUN-Forward: GCTGCTCTGGGAAGTGAGTT
c-JUN-Reverse: TTTCTCTAAGAGCGCACGCA
c-MYC-Forward: GGACCCGCTTCTCTGAAAG
c-MYC- Reverse: GTCGAGGTCATAGTTCCTGTTG
GAPDH-Forward: GAAGGTGAAGGTCGGAGTC
GAPDH-Reverse: GAAGATGGTGATGGGATTTC

### Western Blot

To detect cellular level of target proteins, protein extracted from THCA cells were detected by Western Blot. Lysis buffer consisting of Tris (50 mM, pH7.4), EDTA (1 mM), NaCl (150 mM), 10% Glycerol, 1% Triton, as well as protease/phosphatase inhibitor cocktail (Roche, Basel, Switzerland) was used to extract cell lysates. Bradford assay was performed to determine protein content. Later, we performed SDS-PAGE to separate 30 to 40 μg soluble proteins. Afterwards, electrophoretic transfer of the isolated proteins to PVDF membranes (Millipore, Billerica, MA, USA) was conducted. Primary antibodies utilized in the present study were diluted into 5% nonfat milk as 1:500. Immunoreactive proteins were visualized using EasyBlot ECL kit (Sangon Biotech, China). Gray value of each protein band of western blots picture were analyzed by ImageJ (Rawak Software, Inc. Germany).

### Cell Proliferation Test

Cell proliferation test was performed according to CCK-8 manufacturer’s instruction on day 0, 1, 2, 3, and 4 after transfection (Lot. PJ762, DOJINDO Laboratories).1000 cells were seeded in 96 wells plate and culture overnight. CCK8 reagent was added at the time point and measured by DNM-9602 Microplate Reader (Perlong, Beijing, China).

### Colony Formation Assay

Individual cells were suspended into medium. Each group was inoculated with l0 ml culture medium with 200 cells per dish, and the cells were evenly dispersed by gentle shaking. Routine culture for 3 weeks. We eliminated the medium once there was clone seen within the petri dish, followed by 15 min of 4% paraformaldehyde fixation, 10 min of 0.1% crystal violet staining, PBS washing, and the number of clones was counted.

### Transwell Chamber Assay

After 24 h of starving, logarithmic growth cells were digested the cells the next day, centrifugated, and resuspended, with a final concentration of 2×10^5^/ml. Each well of the Transwell upper chamber was added with 0.2 ml suspension, and the lower chamber was added with 700 ml of precooled DMEM/RPMI 1640 that contained 10% FBS. Thereafter, we cultured cells within the cell incubator under 37°C and 5% CO2 conditions. After 24 h, we removed the Transwell chamber, and the cotton swabs were used to scrape cells within the upper and basement membranes. Afterwards, methanol was used to fix cells for 30 min, followed by 20 min of 0.1% crystal violet staining. Five fields (100×) were randomly selected to count the number of transmembrane cells.

### Wound Healing Assay

Logarithmic growth cells were planted into the 24-well plate when 70% to 80% cell fusion was achieved at 24 h after growth. Used a new 1 ml pipette tip to gently scratch the monolayer. After scraping, wells were washed using the culture medium gently for the removal of detached cells. The wells were supplemented with fresh medium, the cells were cultured for another 48 h and rinsed by 1× PBS twice, followed by 30 min of fixation using 3.7% paraformaldehyde and 30 min of 1% crystal violet staining within the 2% ethanol and photographed with a microscope.

### *In Vivo* Xenograft Model

We obtained twenty 4-week-old BALB/Cnu/nu nude mice (20 g) from Beijing Vital River Laboratory Animal Technology Co., Ltd. and raised them under the pathogen-free conditions. All experimental operations follow the International Laboratory Animal Ethics Convention and comply with relevant national regulations.

We dissolved BCPAPi cells into 200 μl saline at 1×10^6^, followed by subcutaneous injection in nude mice at the right side. Thereafter, we monitored tumor growth at regular intervals. When the tumor is clearly observable, mice were randomly divided into three subgroups with the same number, and received DOX food, normal food with 2 to 4 Da (4) (2,4-Diamino-quinazolines, 25 mg/kg) or normal food every day. Measure the length of the two largest sides of the tumor with a vernier caliper every 3 days, and use the formula V=L×W2×0.5 (L is the length; W is the width) to calculate tumor volume. After 28 days, the transplanted tumor was stripped and weighed.

### Aging-Related β-Galactosidase Staining Assay

Cell Signaling Senescence β-Galactosidase Staining Kit (CST company, USA) was used in β-galactosidase staining and performed according to manual.

### IHC Staning

In this study, IHC staining of the transplanted tumor tissues was performed using the IHC staining step 1 on the Leica Bond-Max/Bond-III automatic immunohistochemical staining machine. Antigen was repaired using the heat-induced epitope repair (HIER) method. The primary antibody: Anti-Ki67 (ab16667) and Anti-p21(ab188224) and secondary antibody: Goat Anti-Rabbit IgG H&L (HRP) (ab97051) were purchased from Abcam.

### Statistical Analysis

Each experiment in the present work was performed in triplicates. Data were expressed in the manner of mean ± SD calculated by STDEV formula in Excel. The significance of all data was estimated by a Tukey’s multiple-comparison test in the ANOVA analysis using the SigmaStat 3.5 software. Importantly, *P* < 0.05 suggested statistical significance.

## Results

### ZNF24 Is the Novel THCA Suppressor Gene With Clinical Relevance

Clinically, the effective treatment options available to THCA patients are very limited. In order to identify functional and important tumor suppressor genes (TSGs), and explore the signal transduction mechanisms as the drug targets for THCA patients. We analyzed the data of THCA in TCGA and found that ZNF24 showed high expression within THCA para-tumoral samples but low within THCA tumor samples (**Figures 1A, B** **)**. In the detection of clinical samples (**Table 1**), we confirmed that ZNF24 mRNA and protein expression within para-carcinoma samples remarkably increased relative to that within tumor samples (**Figures 1C, D** **)**. In order to verify the TSG function of ZNF24, we attempted to ectopic expression of ZNF24 in human THCA cells. As a result, ZNF24 expression within human THCA cells decreased slowly compared with para-carcinoma samples (**Figure 1E**). We selected human THCA cell lines BCPAP and K1/GLAG-66, and constructed these two types of cells to determine the doxycycline (DOX)-induced ZNF24 expression (deemed as BCPAPi and K1/GLAG-66i, separately; **Figure 1F**). As a result, ectopic ZNF24 expression remarkably reduced colony growth and colony formation ability within the 2D-plate of BCPAPi and K1/GLAG-66i cells (**Figures 1G–I**). In addition, ectopic expression of ZNF24 inhibited sphere formation ability of K1/GLAG-66i and BCPAPi cells as well (**Figure 1J**). Taken together, our data suggested that ZNF24 is a novel and clinically relevant THCA TSG.

**Figure 1:** ZNF24 serves as a new suppressor gene of THCA with clinical relevance **(A, B)** mRNA levels of ZNF24 within the GTEX-derived thyroid samples and TCGA-derived THCA samples; **(C)**: mRNA expression of ZNF24 in para-tumoral tissues and in tumor tissues; **(D)**: Western blotting on the ZNF24 level within specific lung tissue samples, T: tumor, N: para-tumor; **(E)**: Western blotting on the ZNF24 level within specific THCA cells **(F)** Impacts of DOX-mediated ZNF24 expression within stable BCPAPi and K1/GLAG-66i cells. Immunoblots that contained specific antibodies were used to analyze specific cells-derived whole-cell lysates; **(G, H)** ZNF24 ectopic expression inhibited K1/GLAG-66i and BCPAPi cells cell viability. The K1/GLAG-66i **(F)** and BCPAPi cells **(G)** (1 × 10^3^) were exposed to 48 h of 1 µg/ml DOX treatment or not, and CCK-8 assay was conducted to detect cell viability at specific time points; **(I)** ZNF24 suppressed the ability of form colonies in BCPAPi and K1/GLAG-66i cells. K1/GLAG-66i and BCPAPi cells were exposed to 10 days of DOX treatment prior to colony formation assay; **(J)** ZNF24 suppressed the ability to form spheres in BCPAPi and K1/GLAG-66i cells. Typical sphere formation image for BCPAPi and K1/GLAG-66i cells (upper), as well as sphere formation statistic image (lower). Values are obtained from three independent assays, while unpaired t-test was used for analysis. Error bars = SD. *P < 0.05, **P < 0.01.

**Table 1:** Patient samples characteristics.

Characteristic	Patients(n=60)
Age, median (interquartile range), y	46 (29-71)
Male, No. (%)	36 (60)
Tumor size, median (interquartile range), cm	1.64(0.43-3.24)
TNM stage, No. (%)	
I	14(23.33)
II	28(46.67)
III	11(18.33)
IV	7(11.67)
Tumor differentiation, No. (%)	
High-moderate	19(31.67)
Low	41(68.33)
Lymph node metastasis, No. (%)	
Positive	8(13.33)
Negative	52(86.67)

### ZNF24 Inhibited K1/GLAG-66i and BCPAPi Cells Invasion and Migration

We than asked how ZNF24 affected THCA cell invasion and migration, Transwell and wound healing assays were carried out. According to **Figures 2A, B**, ectopic expression of ZNF24 significant inhibited K1/GLAG-66i and BCPAPi cell migration compared with contorl group. In addition, ectopic expression of ZNF24 significant inhibited K1/GLAG-66i and BCPAPi cell invasion (**Figure 2C**). Furthermore migration and invasion protein makers: Cox-2, MMP-2, and MMP-9 were significant inhibited by ZNF24 compared with control group (**Figures 2D–F**). Taken together, these data indicated K1/GLAG-66i and BCPAPi cell migration and invasion were inhibited through ectopic expression of ZNF24.

**Figure 2:** ZNF24 inhibited K1/GLAG-66i and BCPAPi cells migration and invasion. **(A–C)** Cell migration and invasion detection by Wound Healing test **(A)** and transwell chamber assay **(B, C)** of K1/GLAG-66i and BCPAPi cells treated without or with DOX (1 µg/ml); **(D)** Cell migration and invasion protein makers expression level detection by Western Blot assay of K1/GLAG-66i and BCPAPi cells treated without or with DOX (1 µg/ml), indicated antibodies were added during Western Blot assay; **(E, F)** Statistical analysis of cell migration and invasion protein makers expression level based on western blot assay result Values are obtained from 3 independent assays, while unpaired t-test was used for analysis. Error bars= SD. *P < 0.05; **P < 0.01.

### Ectopic ZNF24 Expression Led to THCA Cell Aging

TSGs function to suppress tumor genesis through arresting the cell cycle, suppressing cell aging and apoptosis. To detect how ZNF24 performs its its tumor suppressive function, this study examined how the ZNF24 level affected the distribution of cell cycle. As shown in **Figure 3A**, the ZNF24 level resulted in significantly increased G0/G1 cell percentages in K1/GLAG-66i and BCPAPi cells, while the percentage of S phase decreased. We also noticed that K1/GLAG-66i and BCPAPi cells cultivated within the medium that contained DOX showed a flattened, irregular and enlarged morphology (Data unshown), which represented the typical morphology of aging cells. Through the β-galactosidase staining assay, we further confirmed the senescence of K1/GLAG-66i and BCPAPi cells was induced by ZNF24 (**Figure 3B**). In summary, findings in this study suggested that ZNF24 played the TSG role through triggering the aging of THCA cells.

**Figure 3:** Ectopic ZNF24 expression led to THCA cell aging. **(A)** ZNF24 induces G0/G1 cell cycle arrest in K1/GLAG-66i and BCPAPi cells. Cell proportions at G0/G1, S, G2/M phases. BCPAPi and K1/GLAG-66i cell lines were exposed to 3 days of 1 µg/ml DOX treatment or not, the distribution of cell cycle (left) and the related statistics (right) were analyzed by FACS analysis. **(B)** ZNF24 ectopic expression induced senescence of THCA cells. BCPAPi and K1/GLAG-66i cell lines were exposed to 48 h of 1 µg/ml DOX treatment or not, the activity of aging-related β-galactosidase (left) and the related statistics (right) were analyzed to determine the aging cells. Values are obtained from three independent assays, while unpaired t-test was used for analysis. Error bars=SD. *P < 0.05.

### ZNF24 Inhibits the Wnt Signal Transduction Pathway Activation Within BCPAPi Cells by Competitively Binding β-Catenin

In order to find out the precise mechanisms related to the ZNF24-induced aging of THCA cells.Lu et al. reported that Wnt signaling pathway is related to tumor cells senescence (11). We dected the impact of ZNF24 on Wnt signaling pathway in BCPAPi cells, and the qPCR assay result showed that ZNF24 expression significantly downregulated target genes in the typical Wnt signal transduction pathway, such as CCND2, cJUN, C-MYC and AXIN2 (**Figure 4A**). As verified by Western blotting, target genes in the Wnt signaling pathway were down-regulated at protein level (**Figure 4B**). As β-catenin exerts a vital part in representative Wnt signal transduction activity, we speculated that ZNF24 interacts with β-catenin. To verify this hypothesis, we performed immunoprecipitation (IP) in DOX treated BCPAPi cells. According to **Figure 4C**, ectopic over-expression of ZNF24 predicted β-catenin expression within BCPAPi cells. Generally speaking, β-catenin proteins are stably accumulated within cytoplasm, which then experience nuclear imports to form complexes with TCF1/LEF1, which activates Wnt signaling pathway [33]. According to Co-IP assays, BCPAPi cells exposed to DOX had effectively inhibited LEF1 or TCF1 knockdown by endogenous β-catenin. Co-IP assay demonstrated that ectopic ZNF24 expression remarkably decreased the endogenous β-catenin ability of pulling down LEF1 or TCF in BCPAPi cells (**Figure 4D** **)**. In conclusion, findings in this work suggested that ZNF24 suppressed the formation of β-catenin functional complex with cofactors including LEF1/TCF1 by competitively binding β-catenin, which inhibited the Wnt signaling pathway.

**Figure 4:** ZNF24 inhibits the activation of Wnt signaling pathway in BCPAPi cells by competitively binding β-catenin. **(A)** ZNF24 inhibits Wnt signaling pathway traget genes mRNA expression. BCPAPi cells (2 × 10^5^) were subjected to 48 h of 1 µg/ml DOX treatment or not, then qPCR was conducted to extract total RNA; **(B)** Wnt signaling pathway traget genes protein expression level detection by Western Blot assay of BCPAPi cells treated without or with DOX (1 µg/ml), indicated antibodies were added during Western Blot assay. **(C)** Endogenous ZNF24 is associated with β-catenin within the BCPAPi cell line. CoIP assays were carried out using anti-β-catenin or anti-ZNF24, then immunoblots that contained specific antibodies were used to analyze whole-cell lysate and immunoprecipitates (input). **(D)** ZNF24 diminish the interaction between β-catenin and TCF1 or LEF1. 2.5 g plasmids were used to transfect 293T cells (2 × 10^6^). CoIP and immunoblot assays were carried out using specific antibodies. Values are obtained from 3 independent assays, while unpaired t-test was used for analysis. Error bars=SD. *P < 0.05, **P < 0.01.

To further conformed the ZNF24 induced BCPAPi cells senescence through regulating Wnt signaling pathway. Inhibitors of the Wnt signal transduction pathway were measured: ICG001 on BCPAPi cells. As shown in **Figures 5A, B**, ICG001 has a similar effect to ectopic ZNF24 expression, and it remarkably reduced colony formation within 2D-plate in BCPAPi cells. In addition, ICG001 significantly increased senescence BCPAPi cells number (**Figure 5C**). Next, we verified whether ZNF24 induced BCPAPi cells senescence through interacting with β-catenin. We overexpressed β-catenin in BCPAPi cells (**Figure 5D**).

**Figure 5:** β-catenin reverse the ZNF24 effect of BCPAPi cells. **(A, B)** Cell viability and colony forming dectection of BCPAPi cells without or with DOX (1 µg/ml) or ICG001 (0.1 μg/ml) treatment. **(C)** ICG001 induces senescence of BCPAPi cells. BCPAPi cells without or with DOX (1 µg/ml) or ICG001 (0.1 μg/ml) treatment for 48 h, later the aging cells were measured through activity of aging-related β-galactosidase (left) and the corresponding statistics (right). **(D)** β-catenin expression level detection by Western Blot assay. 0.1 μg β-catenin expression plasmids were transfected into BCPAPi cells (1 × 10^4^), followed by DOX (1 µg/ml of DOX treatment or not, indicated antibodies were added during Western Blot assay. **(E, F)** Cell viability and colony forming dectection of BCPAPi cells. 0.1 μg β-catenin expression plasmids were transfected into BCPAPi cells (1 × 10^4^), followed by 1 µg/ml of DOX treatment or not. **(G)** BCPAPi cells (1 × 10^4^) were transfected with β-catenin expression plasmid (0.1 μg), followed by 1 µg/ml of DOX treatment or not. The aging cells were measured through the activity of aging-related β-galactosidase (left) and the corresponding statistics (right). Values are obtained from three independent assays, while unpaired t-test was used for analysis. Error bars=SD. *P < 0.05, ***P < 0.001.

We found out that the ectopic expression of ZNF24 inhibition of BCPAPi cells growth rate and colony forming ability was reversed by overexpressing β-catenin (**Figures 5E, F** **)**. Further more, this reverse effect casued by overexpressing β-catenin was observed in ZNF24 induced BCPAPi cells senescence condition as well (**Figure 5G**). To sum up, these results indicated that ZNF24 induced BCPAPi cells senescence through regulating Wnt signaling pathway.

### ZNF24 and 2,4-Da Inhibited THCA Xenografted Tumors Growth in Nude Mice

For investigating the effect of ZNF24 on THCA xenografted tumors in nude mice. BCPAPi cells were subjected to subcutaneous inoculation into nude mice, which were then randomly treated with medium that contained DOX, Wnt signaling pathway inhibitor: 2,4-Da or normal food (control diet). Both ectopic expression of ZNF24 and 2,4-Da significantly shrinked xenografted tumors volume and weight in comparation to the control diet group (**Figures 6A, B, D** **)**. In addition, the DOX and 2,4-Da have non-toxic effect of mice, as evidenced by the unchanged mouse weight in the experimental process (**Figure 6E**). The DOX treatment significantly inhibited ZNF24 mRNA expression level (**Figure 6C**) and ZNF24 protein expression level (**Figure 6F**). Furthermore, IHC staining assay results showed that both ectopic expression of ZNF24 decreased the proliferation marker Ki-67 protein level relative to control diet group, and the combined treatment of ZNF24 and 2,4-Da had a more significant effect on tumor inhibition (**Figure 6G**). As expected, DOX significantly increased the expression of p21(a marker of senescence) in xenografted tumors (**Figure 6H**). Taken together, our data demonstrated both ectopic expression of ZNF24 and 2,4-Da could inhibited THCA xenografted tumors growth in nude mice.

**Figure 6:** ZNF24 and 2,4-Da inhibited THCA xenografted tumors growth in nude mice. **(A, B, D)** The growth and weight of DOX or 2,4-Da exposed tumor samples was significantly inhibited relative to controls. We measured tumor growth at intervals of 2 days by measuring its diameter with Vernier caliper. **(C)** The Real Time PCR analysis of ZNF24 on ex vivo tumor extracts. **(E)** 2,4 Dia or DOX made no difference to the mouse body weight measured at intervals of 5 days. **(F)** Protein expression level of ZNF24 of THCA xenografted tumors of nude mice treated with DOX (DOX+) or without DOX (DOX-). **(G, H)** IHC staining of THCA xenografted tumors of nude mice treated with DOX (DOX+), DOX+2,4-Da or without DOX (DOX-), indicated antibodies were added during IHC staining assay. Values are obtained from three independent assays, while unpaired t-test was used for analysis. Error bars=SD. *P < 0.05; **P < 0.01; ***P < 0.001.

## Discussion

Despite significant advances in clinical treatment of THCA in recent years, it remains lacking of the effective treatment options available to THCA patients (15–17). The difficulties in the treatment of patients with THCA stem from our limited understanding of molecular mechanism of tumor occurrence, and this provides a new research direction recently (18–21). Elucidating the molecular mechanism controlling tumorigenesis of THCA is of great importance. This study identified tumor suppressor inducing THCA tumor cells senescence module not discovered before, which might serve as the therapeutic opportunity for ZNF24 deficient THCA patients.

In this study, the high ZNF24 expression was detected within para-carcinoma samples, while low expression was detected in THCA tumor tissues in all THCA patients and demonstrated tumor suppressor function of ZNF24 in THCA. Of note, several recent studies have shown that ZNF24 is the tumor suppressor gene of HCC (12, 22). This indicated that elucidating the molecular mechanism underlying ZNF24 tumor suppressor function in THCA had clinical significance.

As an important transcription factor in the classic Wnt signal transduction pathway, β-catenin is recognized as the oncogene (23–25). Due to its importance, studies have been suggested that β-catenin can promote tumor development, and the therapeutic effects of drugs targeting β-catenin in preclinical tumor models are suggested (26–29). This work identified a previously unnoticed tumor suppressor inducing THCA tumor cells senescence mechanism,which was that ZNF24 suppressed the formation of functional complex of β-catenin with cofactors such as LEF1/TCF1 by competitively binding β-catenin. which inhibitd the Wnt signaling pathway. This competitively binding effect inhibited Wnt signaling pathway activition resulting in THCA cells senescence. And the ZNF24 inducing senescence inhibited THCA tumorigenesis and invasion. Our study suggested that THCA patients with ZNF24 deficiency were associated with up-regulated typical Wnt signal transduction activity. According to our preclinical study, 2,4-Dia, a Wnt signaling pathway inhibitor, is safe and effective (30). This may be a therapeutic opportunity for ZNF24 deficient THCA patients.

In conclusion, our current study found out the tumor suppressor function of ZNF24 in THCA and demonstrated its competitively binding effect inhibited Wnt signaling pathway activition resulting in THCA cells senescence. Considering that ZNF24 deficiency is highly prevalent in THCA cases, this study may offer a therapeutic opportunity for ZNF24 deficient THCA patients.

## Data Availability Statement

The original contributions presented in the study are included in the article/supplementary material. Further inquiries can be directed to the corresponding author.

## Ethics Statement

All experimental protocols were approved by the Institutional Committee for Animal Care and Use at Shenzhen University. All animal work was performed in accordance with the approved protocol.

## Author Contributions

JX mainly participated in literature search, study design, writing, and critical revision. LZ and YW mainly participated in data collection, data analysis, and data interpretation. PJ organized the pathological information form, conducted the PCR and ICH, drafted schametic diagram and made important contributions to revising the manuscript and responding to the reviewer’s questions. All authors contributed to the article and approved the submitted version.

## Funding

This work was supported by funding from the National Natural Science Foundation of China (No. 81903412 awarded to JX).

## Conflict of Interest

Author PJ was employed by company Shenzhen RealOmics (Biotech) Co., Ltd.

The remaining authors declare that the research was conducted in the absence of any commercial or financial relationships that could be construed as a potential conflict of interest.

## References

[1] SiegelRLMillerKDJemalA. Cancer Statistics, 2019. CA Cancer J Clin (2019) 69:7–34. 10.3322/caac.21551 30620402

[2] Bibbins-DomingoKGrossmanDCCurrySJBarryMJDavidsonKWDoubeniCA. Screening for Thyroid Cancer US Preventive Services Task Force Recommendation Statement. Jama-Journal Am Med Assoc (2017) 317:1882–7. 10.1001/jama.2017.4011 28492905

[3] PellegritiGFrascaFRegalbutoCSquatritoSVigneriR. Worldwide Increasing Incidence of Thyroid Cancer: Update on Epidemiology and Risk Factors. J Cancer Epidemiol (2013) 2013:965212. 10.1155/2013/965212 23737785PMC3664492

[4] ChenZVenkatesanAMDehnhardtCMDos SantosODelos SantosEAyral-KaloustianS. 2,4-Diamino-Quinazolines as Inhibitors of aBeta-Catenin/Tcf-4 Pathway: Potential Treatment for Colorectal Cancer. Bioorganic medicinal Chem Lett (2009) 19:4980–3. 10.1016/j.bmcl.2009.07.070 19640711

[5] XingM. Molecular Pathogenesis and Mechanisms of Thyroid Cancer. Nat Rev Cancer (2013) 13:184–99. 10.1038/nrc3431 PMC379117123429735

[6] VellaVMalaguarneraR. The Emerging Role of Insulin Receptor Isoforms in Thyroid Cancer: Clinical Implications and New Perspectives. Int J Mol Sci (2018) 19:3814. 10.3390/ijms19123814 PMC632133030513575

[7] VellaVPuppinCDamanteGVigneriRSanfilippoMVigneriP. Deltanp73alpha Inhibits PTEN Expression in Thyroid Cancer Cells. Int J Cancer (2009) 124:2539–48. 10.1002/ijc.24221 19173293

[8] Sastre-PeronaASantistebanP. Role of the Wnt Pathway in Thyroid Cancer. Front Endocrinol (Lausanne) (2012) 3:31. 10.3389/fendo.2012.00031 22645520PMC3355838

[9] Garcia-RostanGCampRLHerreroACarcangiuMLRimmDLTalliniG. Beta-Catenin Dysregulation in Thyroid Neoplasms: Down-Regulation, Aberrant Nuclear Expression, and CTNNB1 Exon 3 Mutations are Markers for Aggressive Tumor Phenotypes and Poor Prognosis. Am J Pathol (2001) 158:987–96. 10.1016/S0002-9440(10)64045-X PMC185033611238046

[10] Garcia-RostanGTalliniGHerreroAD’AquilaTGCarcangiuMLRimmDL. Frequent Mutation and Nuclear Localization of Beta-Catenin in Anaplastic Thyroid Carcinoma. Cancer Res (1999) 59:1811–5.10213482

[11] LuFZhouQLiuLZengGDCiWMLiuWT. A Tumor Suppressor Enhancing Module Orchestrated by GATA4 Denotes a Therapeutic Opportunity for GATA4 Deficient HCC Patients. Theranostics (2020) 10:484–97. 10.7150/thno.38060 PMC692998431903133

[12] LiuXYGeXXZhangZZhangXWChangJJWuZ. Microrna-940 Promotes Tumor Cell Invasion and Metastasis by Downregulating ZNF24 in Gastric Cancer. Oncotarget (2015) 6:25418–28. 10.18632/oncotarget.4456 PMC469484126317898

[13] LiuGJiangSWangCJiangWLiuZLiuC. Zinc Finger Transcription Factor 191, Directly Binding to Beta-Catenin Promoter, Promotes Cell Proliferation of Hepatocellular Carcinoma. Hepatology (2012) 55:1830–9. 10.1002/hep.25564 22213192

[14] ZouFWYangSZLiWYLiuCYLiuXHHuCH. Circrna_001275 Upregulates Wnt7a Expression by Competitively Sponging Mir3703p to Promote Cisplatin Resistance in Esophageal Cancer. Int J Oncol (2020) 57:151–60. 10.3892/ijo.2020.5050 PMC725246232319613

[15] KreugerETrommlerB. Thyroid Cancer: Diagnosis, Treatment and Prognosis . New York: Nova Biomedical (2013).

[16] KreugerETrommlerB. Thyroid Cancer : Diagnosis, Treatment and Prognosis. In: . Cancer Etiology , Diagnosis, and Treatments. New York: Nova Biomedical (2013). p. 1 online resource.

[17] ZhangLLuoHWangLLiuYZhuJ. Diagnostic and Prognostic Value of Preoperative Systemic Inflammatory Markers in Anaplastic Thyroid Cancer. J Surg Oncol (2020) 122:897–905. 10.1002/jso.26089 32596828

[18] Van NostrandD. Thyroid Cancer : A Guide for Patients. 2nd ed. Pasadena, MD: Keystone Press (2010).

[19] Van NostrandDBloomGWartofskyL. Thyroid Cancer : A Guide for Patients. Baltimore, MD: Keystone Press (2004).

[20] WartofskyL. Thyroid Cancer : A Comprehensive Guide to Clinical Management. Totowa, N.J: Humana Press (2000).10975951

[21] JosephFGRubtsovDDavorenP. Appropriateness of Ultrasound Imaging for Thyroid Pathology, the Standard of Radiology Reporting on Thyroid Nodules and the Detection Rates of Thyroid Malignancy: A Tertiary Centre Retrospective Audit. Internal Med J (2020) 50:732–40. 10.1111/imj.14401 31180168

[22] HuangXJLiuNXXiongX. ZNF24 is Upregulated in Prostate Cancer and Facilitates the Epithelial-to-Mesenchymal Transition Through the Regulation of Twist1. Oncol Lett (2020) 19:3593–601. 10.3892/ol.2020.11456 PMC711515832269634

[23] DebebeAMedinaVChenCYMahajanIMJiaCFuD. Wnt/β-catenin activation and macrophage induction during liver cancer development following steatosis. Oncogene (2017) 36(43):6020–9. 10.1038/onc.2017.207 PMC566631728671671

[24] ChenYLiYWangXQMengYZhangQZhuJY. Phenethyl Isothiocyanate Inhibits Colorectal Cancer Stem Cells by Suppressing Wnt/Beta-Catenin Pathway. Phytotherapy Res (2018) 32:2447–55. 10.1002/ptr.6183 30159926

[25] SalzetM. β-Catenin knockdown promotes NHERF1-mediated survival of colorectal cancer cells: implications for a double-targeted therapy. Oncogene (2018) 37:3301–16. 10.1038/s41388-018-0170-y PMC600234429551770

[26] JeongWJRoEJChoiKY. Interaction between Wnt/β-catenin and RAS-ERK pathways and an anti-cancer strategy via degradations of β-catenin and RAS by targeting the Wnt/β-catenin pathway. npj Precision Oncology (2018) 2(1)5. 10.1038/s41698-018-0049-y PMC587189729872723

[27] CuiJJJiangWHWangSYWangLWXieKP. Role of Wnt/Beta-Catenin Signaling in Drug Resistance of Pancreatic Cancer. Curr Pharm Design (2012) 18:2464–71. 10.2174/13816128112092464 22372504

[28] JiangHLJiangLMHanWD. Wnt/Beta-Catenin Signaling Pathway in Lung Cancer Stem Cells is a Potential Target for the Development of Novel Anticancer Drugs. J Buon (2015) 20:1094–100.26416062

[29] JungYSParkJI. Wnt Signaling in Cancer: Therapeutic Targeting of Wnt Signaling Beyond Beta-Catenin and the Destruction Complex. Exp Mol Med (2020) 52:183–91. 10.1038/s12276-020-0380-6 PMC706273132037398

[30] ChenZCVenkatesanAMDehnhardtCMDos SantosODelos SantosEAyral-KaloustianS. 2,4-Diamino-Quinazolines as Inhibitors of Beta-Catenin/Tcf-4 Pathway: Potential Treatment for Colorectal Cancer. Bioorganic Medicinal Chem Lett (2009) 19:4980–3. 10.1016/j.bmcl.2009.07.070 19640711

